# Efficacy and Safety of Intravitreal Injection of Triamcinolone Acetonide and Conbercept for Intraocular Lens after Cataract Surgery

This article has been retracted.

**DOI:** 10.1155/2022/5606343

**Published:** 2022-05-25

**Authors:** Bin Tang, Xiaoxuan Wang, Yi Luo, Zhi Li, Yannan He

**Affiliations:** ^1^Ophthalmology Department, Chongqing Red Cross Hospital (Jiangbei District People's Hospital), Chongqing 400020, China; ^2^Hebei Eye Hospital, Hebei Provincial Key Laboratory of Ophthalmology, Hebei Provincial Clinical Research Center for Eye Diseases, Xingtai, Hebei 054000, China; ^3^Ophthalmology Department, Chongqing Jiulongpo District Second People's Hospital, Chongqing 400020, China

## Abstract

**Objective:**

To investigate the effect of intravitreal injection of triamcinolone acetonide and conbercept on the efficacy and safety of diabetic macular edema (DME) after cataract intraocular lens (IOL) surgery.

**Methods:**

A total of 350 patients with cataract complicated with diabetic macular edema in our hospital from January 2017 to July 2021 were randomly divided into conbercept group and triamcinolone acetonide group. Patients in the conbercept group were given intravitreal injection of conbercept during IOL surgery, and patients in the triamcinolone acetonide group were given injection of triamcinolone acetonide during surgery.

**Results:**

Three months after treatment, the best-corrected visual acuity of the two groups was significantly higher than before, the corrected visual acuity of the conbercept group was more significant than the triamcinolone acetonide group, and the intraocular pressure of the triamcinolone acetonide group was higher than the conbercept group. The foveal thickness and macular volume were significantly reduced in both groups, and was reduced more in the conbercept group than in the triamcinolone acetonide group. The contents of VEGF, SDF-1, and IL-6 in both groups were significantly decreased, and the decrease was more significant in the conbercept group than in the triamcinolone acetonide group. The patients with elevated intraocular pressure, headache and vomiting, orbital swelling pain, eye swelling pain, and eye pain in the triamcinolone acetonide group were significantly higher than those in the conbercept group (*P* < 0.05).

**Conclusions:**

Conbercept and triamcinolone acetonide has a good therapeutic effect on DME in pseudophakic eyes after cataract IOL surgery, which can reduce the degree of macular edema and improve the visual function. However, the therapeutic effect of injection therapy with conbercept is safe, the prognosis is better, and the complication rate is low.

## 1. Introduction

In China, the incidence of diabetes is increasing. A state of hyperglycemia will lead to a series of complications in patients, such as cardiovascular disease and eye diseases. [1, 2]. Cataract is one of the most common ocular complications in diabetic patients, more occurring in middle-aged and elderly diabetic patients, often resulting in decreased visual acuity [3], opacity, and haziness [4], and has a high rate of blindness [5]. There are many factors leading to cataract such as ocular aging and nutritional disorders, immune abnormalities, and genetics. [6–8]. With the continuous development of cataract surgery technology, implantation of IOL has become a commonly treatment for cataract [9]. However, surgery can induce serious mechanical damage to the eye and foreign body reactions. Some residual lens cortex will stimulate the cells around the eye to secrete arachidonic acid, phospholipase, and other substances. Arachidonic acid synthesizes prostaglandins under the action of cyclooxygenase, resulting in the damage of blood-retinal barrier and impaired function [10]. After the damage of blood-retinal barrier, a series of fundus changes will gradually appear. Under the combined action of ischemia and increased inflammatory secretions, the macular volume increases, the blood vessels in the macular area increase, and the permeability of the surrounding capillary osmotic pressure changes increases [6], which makes the protein molecules, water, and other components in the blood easily penetrate out through the vascular wall and effusion under the retina, causing retinal thickening, and the fibers in the macula are arranged in a radial pattern [11]. When the accumulated fluid reaches a certain amount, it will cause diabetic macular edema, affecting the visual recovery of patients [12].

At present, intravitreal injection of conbercept or triamcinolone acetonide ophthalmic is mostly used to reconstruct the blood-retinal barrier in patients with diabetic macular edema in clinical practice [13]. Triamcinolone acetonide is an adrenocortical hormone drug, which has the effects of local, antiallergic, inhibiting neovascularization and cell proliferation, reducing vascular permeability, and stabilizing the blood-retinal barrier, and can improve macular edema [14, 15]. Corbercept, as an intravitreal vascular endothelial growth factor (VEGF) inhibitor, has good clinical efficacy in the treatment of diseases such as diabetic macular edema [16, 17].

In this study, we aimed to explore the therapeutic efficacy and safety of intravitreal injection of triamcinolone acetonide and conbercept in patients with DME in pseudophakic eyes after cataract IOL surgery and provide more reference for clinical practice.

## 2. Materials and Methods

### 2.1. Study Design and Participants

A total of 350 cataract patients with DME in our hospital from January 2017 to July 2021 were enrolled in for this retrospective study. There were 176 patients in the conbercept group, 94 males and 82 females, aged 50–80 years; 174 patients in the triamcinolone acetonide group, 85 males and 89 females, aged 48–83 years. There was no significant difference in the baseline data of the patients (*P* > 0.05). Informed consent was obtained from all patients. The study was approved by the Ethics Committee of Chongqing Red Cross Hospital (No.CRH2171). All participants underwent a complete medical history and clinical examination.

### 2.2. Observation Indicators

1. The best-corrected visual acuity and intraocular pressure were measured by international standard visual acuity chart and Goldmann tonometer before treatment and 3 months after treatment in both groups. The normal intraocular pressure value is generally 10–21 mmHg.
2. Foveal thickness and macular volume were measured by optical coherence tomography before treatment and 3 months after treatment in both groups.
3. 3 mL fasting peripheral venous blood was collected from patients in both groups before and after treatment, and after centrifugation at 3000 r/min for 15 min, the content of VEGF and stromal cell-derived factor-1 (SDF-1) was measured by the immunohistochemistry assay and enzyme-linked immunosorbent assay, respectively. The content of interleukin-6 (IL-6) was determined by the cell proliferation assay.
4. Complications after treatment were observed in both groups.

### 2.3. Inclusion and Exclusion Criteria

Inclusion criteria are as follows: (1) patients who meet the diagnostic criteria of cataract with diabetic macular edema. (2) No history of ocular diseases such as glaucoma, high hyperopia or myopia, and maculopathy. (3) Patients and their families understand the study details, agree to participate in this experiment, and sign an informed consent form. (4) No serious heart, liver, kidney dysfunction or malignant tumors, and other diseases.

Exclusion criteria are as follows: (1) patients who were unable to undergo intraocular lens insertion surgery due to special reasons such as posterior capsule rupture and zonular disconnection. (2) Patients who have taken immunosuppressive or anti-inflammatory drugs within three months before treatment. (3) Patients who were hypersensitivity to triamcinolone acetonide and conbercept. (4) Patients with incomplete relevant clinical data.

### 2.4. Statistical Analysis

The SPSS 25.0 statistical software was used to analyze the data. The clinical data (measurement data) were expressed as mean ± standard deviation (*x* ± *S*). One-way analysis of variance was used to compare between groups. Paired *t*-test was performed for intragroup comparison, independent sample *t*-test was performed for intergroup comparison, enumeration data were expressed as rate (%), *χ*2 test was performed, and *P* < 0.05 was considered statistically significant.

## 3. Results

There were 176 patients in the conbercept group, 94 males and 82 females, aged 50–80 years, with an average age of 63.26 ± 4.87 years and BMI 27.63 ± 1.09; 174 patients in the triamcinolone acetonide group, 85 males and 89 females, aged 48–83 years, with an average age of 62.75 ± 4.65 years and BMI: 25.31 ± 1.15. There was no significant difference in the baseline data of patients (*P* > 0.05, Table 1).

### 3.1. Comparison of Best-Corrected Visual Acuity and Intraocular Pressure before and after Treatment

Before treatment, the best-corrected visual acuity was low and the intraocular pressure was within the normal range in both groups, and there was no significant difference (*P* > 0.05). After treatment, the best-corrected visual acuity of the two groups was significantly higher than before treatment. The corrected visual acuity of the conbercept group was more significant than the triamcinolone acetonide group (*P* < 0.05). The intraocular pressure of the conbercept group was not significantly changed compared with before treatment (*P* > 0.05), and it was significant increase in the triamcinolone acetonide group before treatment (*P* < 0.05), intraocular pressure was significant higher in the triamcinolone acetonide group than conbercept group (*P* < 0.05) (see details in Table 2).

### 3.2. Comparison of Foveal Thickness and Partial Macular Volume before and after Treatment

Before treatment, the foveal thickness and macular volume were bigger in both groups (*P* > 0.05). After treatment, foveal thickness and macular volume were significantly reduced in both groups, the reduction was more significant in the conbercept group than in the triamcinolone acetonide group (*P* < 0.05) (see details in Table 3).

### 3.3. Comparison of VEGF, SDF-1, and IL-6 Levels before and after Treatment

Before treatment, there was no significant difference in the contents of VEGF, SDF-1, and IL-6 between the two groups (*P* > 0.05). Three months after treatment, the contents of VEGF, SDF-1, and IL-6 in both groups were significantly decreased compared with before treatment, the decrease is more significant in the conbercept group than in the triamcinolone acetonide group (*P* < 0.05, Table 4).

### 3.4. Incidence of Complications within 2 months after Injection Therapy

There was no significant difference in the incidence of conjunctival congestion, ocular phobia, ocular easy lacrimation, ocular foreign body sensation corneal edema, and osterior subcapsular opacification between the conbercept group and the triamcinolone acetonide group (*P* > 0.05). The incidence of elevated intraocular pressure, headache and vomiting, orbital pain, eye swelling and pain, and eye pain in the triamcinolone acetonide group were significantly higher than that in the conbercept group (*P* < 0.05, Table 5).

## 4. Discussion

The incidence of diabetic macular edema has gradually increased in recent years, and the untimely treatment will cause a serious burden to families and society [18]. VEGF is a powerful angiogenic growth factor found ubiquitously in neovascular endothelial cells. It can induce vascular endothelial cell division, proliferation, enhance vascular permeability. which a risk factor for the development of DME by aggravating subretinal fluid accumulation and exudation [19, 20]. Some studies have found that the expression of IL-6, a chronic inflammatory factor, in the aqueous humor of DME patients is higher. IL-6 can induce increased VEGF expression and further induce the leakage of blood vessels [21]. VEGF can promote the synthesis of SDF-1 and participate in retinal neovascularization together, and SDF-1 is a chemokine protein with chemotactic cell growth and proliferation and expressed in various tissues such as the eye, which can induce an inflammatory response, and closely related to the condition of DME [22, 23]. Triamcinolone acetonide has a strong antiallergic effect and lasting for a long time. After intravitreal injection, it can block the proliferation of endothelial cells and angiogenesis, achieving the effect of treating fundus vascular diseases and the best-corrected visual acuity of patients [24, 25]. In addition, its action inhibits the production of prostaglandins, downregulates VEGF expression, and has a synergistic effect with conbercept [26]. Conbercept can block the activation of VEGF and SDF-1 receptors by binding to the receptors of VEGF and SDF-1, prevent the expression of VEGF and SDF-1 in cells, and indirectly reduce the expression of IL-6 [27]. Eventually, it reduces the expression of VEGF, SDF-1, and IL-6, inhibits endothelial cell proliferation and angiogenesis, and prevents increased foveal thickness and increased macular partial size in patients [28, 29].

This study showed that three months after treatment, the best-corrected visual acuity of the two groups was significantly higher than before treatment, the corrected visual acuity in the conbercept group was more significant than that in the triamcinolone acetonide group, and the intraocular pressure in the triamcinolone acetonide group was higher than that in the conbercept group. These results indicate that conbercept and triamcinolone acetonide can effectively treat diabetic macular edema, improve the patient's vision, and restore the patient's visual acuity level, but the triamcinolone acetonide injection therapy can lead to increased intraocular pressure in patients. Compared with those before treatment, the foveal thickness and macular volume were significantly reduced in both groups, and the reduction was more significant in the conbercept group than that in the triamcinolone acetonide group (*P* < 0.05). Three months after treatment, the contents of VEGF, SDF-1, and IL-6 in both groups were significantly decreased compared with those before treatment, and the conbercept group was decrease more significant than the triamcinolone acetonide group (*P* < 0.05). It shows that conbercept and triamcinolone acetonide can improve the retinal status of patients by reducing the contents of VEGF, CDF-1, and IL-6, help to reduce the foveal thickness and macular volume. It is worthy of being widely popularized in the clinical application. The comparison of the incidence of complications after treatment between the two groups showed that the incidence of elevated intraocular pressure, headache and vomiting, orbital swelling pain, eye swelling pain and eye pain in the triamcinolone acetonide group were significantly higher than those the compassionate group (*P* < 0.05); there was no significant difference in the incidence of conjunctival congestion, eye fear, eye easy lacrimation, foreign body sensation in the eye, corneal edema, and posterior subcapsular opacification between the two groups. Studies have shown that headache, vomiting, orbital swelling pain, eye swelling and pain, and eye pain are related to elevated intraocular pressure. Therefore, close attention should be paid to the patient's blood pressure during treatment with triamcinolone acetonide injection. Intravitreal injection of triamcinolone acetonide has low safety for the treatment of DME and high incidence of complications after treatment.

In summary, intravitreal injection of conbercept and triamcinolone acetonide has a good therapeutic effect on diabetic macular edema in pseudophakic eyes after cataract surgery, relieving the intravitreal inflammatory response, reducing the degree of macular edema and improving the visual function of patients by reducing the contents of VEGF, CDF-1, and IL-6. However, compared with triamcinolone acetonide, the use of conbercept injection therapy has more considerable safety, better prognosis, reduced the incidence of postoperative complications, and is conducive to improving the quality of life of patients.

## Figures and Tables

**Table 1:** Baseline characteristics.

	Conbercept group (*N* = 176)	Triamcinolone acetonide group (*N* = 174)
Gender (male/female, case)	60/49	50/54
Age (*x* ± *S*, years)	63.26 ± 4.87	62.75 ± 4.65
Weight (kg)	60.42	60.71
BMI (*x* ± *S*, kg/m2)	27.63 ± 1.09	25.31 ± 1.15
Eye disease type (binocular/monocular)	55/54	48/56
Hospital stay (months)	1.75 ± 0.65	1.89 ± 0.47

**Table 2:** Comparison of best-corrected visual acuity and intraocular pressure before and after treatment.

Group	Best-corrected visual acuity (logMAR)		Intraocular pressure (mmHg)	
	Before treatment	3 months after treatment	Before treatment	3 months after treatment
Conbercept group (*N* = 176)	0.37 ± 0.03^a^	0.87 ± 0.23	15.37 ± 2.01	15.29 ± 2.41
Triamcinolone acetonide group (*N* = 174)	0.36 ± 0.05^a^	0.76 ± 0.31	15.40 ± 2.16^a^	16.54 ± 4.96
T	1.779	2.950	0.105	2.356
*P* value	0.077	0.004	0.916	0.019

Compared with pretreatment, ^a^*P* < 0.05.

**Table 3:** Comparison of partial macular volume of foveal thickness before and after treatment.

Group	Foveal thickness (*μ*m)		Macular volume (*μ*m3)	
	Before treatment	3 months after treatment	Before treatment	3 months after treatment
Conbercept group (*N* = 176)	586.42 ± 134.21 a	253.87 ± 80.53	6.45 ± 0.76^a^	4.85 ± 0.03
Triamcinolone acetonide group (*N* = 174)	587.19 ± 136.32 a	294.15 ± 81.66	6.44 ± 0.24^a^	4.82 ± 0.10
T	0.042	3.624	0.128	2.994
*P* value	0.967	<0.001	0.898	0.003

Compared with pretreatment, ^a^*P* < 0.05.

**Table 4:** Comparison of VEGF, CDF-1, and IL-6 levels before and after treatment.

Group	VEGF		SDF-1		IL-6	
	Before treatment	3 months after treatment	Before treatment	3 months after treatment	Before treatment	3 months after treatment
Conbercept group (*N* = 176)	312.46 ± 40.88^a^	180.43 ± 29.01	903.46 ± 65.25^a^	485.23 ± 83.55	13.17 ± 3.01^a^	9.04 ± 3.64
Triamcinolone acetonide group (*N* = 174)	310.87 ± 45.25^a^	206.91 ± 19.87	911.64 ± 60.61^a^	511.72 ± 78.56	12.56 ± 2.74^a^	9.92 ± 2.66
T	0.269	7.736	0.947	2.381	1.544	2.007
*P* value	0.788	<0.001	0.345	0.018	0.124	0.046

Compared with that before treatment, ^a^*P* < 0.05.

**Table 5:** Comparison of incidence rate of postoperative complications (*n* (%)).

Item	Conbercept group (*n* = 176)	Triamcinolone acetonide group (*n* = 174)	Χ2	*P* value
Conjunctival hyperemia (mild/moderate/severe, cases)	68/20/0	79/25/0	0.046	0.813
Eye phobia (case (%))	19 (0.11)	18 (0.10)	0.019	0.981
Eyes with lacrimation (case (%))	16 (0.09)	14 (0.08)	0.122	0.727
Foreign body sensation in eyes (case (%))	14 (0.08)	16 (0.09)	0.172	0.678
Eye pain (case (%))	16 (0.09)	28 (0.16)	3.902	0.048
Corneal edema (case (%))	17 (0.10)	11 (0.06)	1.324	0.250
Posterior subcapsular opacification (case (%))	16 (0.09)	23 (0.13)	1.505	0.220
Intraocular pressure increased (case (%))	10 (0.06)	77 (0.44)	69.691	<0.001
Eye swelling (case (%))	23 (0.13)	56 (0.32)	18.294	<0.001
Orbital pain (case (%))	12 (0.07)	25 (0.14)	5.275	0.022
Headache and vomiting (case (%))	14 (0.08)	26 (0.15)	4.221	0.040

## Data Availability

The data used to support the findings of this study are available from the corresponding author upon request.
